# Lumbar Intervertebral Disc Degeneration Does Not Affect Muscle Synergy for Rowing Activities

**DOI:** 10.1155/2021/6651671

**Published:** 2021-02-15

**Authors:** Chie Sekine, Naoto Matsunaga, Yu Okubo, Mika Hangai, Koji Kaneoka

**Affiliations:** ^1^Department of Physical Therapy, Niigata University of Health and Welfare, 1398 Shimami-cho, Kita-ku, Niigata City, Niigata 950-3198, Japan; ^2^General Education Core Curriculum Division, Seigakuin University, 1-1 Tosaki, Ageo City, Saitama 362-8585, Japan; ^3^School of Physical Therapy, Faculty of Health and Medical Care, Saitama Medical University, 1397-1 Yamane, Hidaka City, Saitama 350-1241, Japan; ^4^Medical Center, Japan Institute of Sports Sciences, 3-15-1 Nishigaoka, Kita-ku, Tokyo 115-0056, Japan; ^5^Faculty of Sport Sciences, Waseda University, 2-579-15 Mikajima, Tokorozawa City, Saitama 359-1192, Japan

## Abstract

Rowers with disc degeneration may have motor control dysfunction during rowing. This study is aimed at clarifying the trunk and lower extremity muscle synergy during rowing and at comparing the muscle synergy between elite rowers with and without lumbar intervertebral disc degeneration. Twelve elite collegiate rowers (with disc degeneration, *n* = 6; without disc degeneration, *n* = 6) were included in this study. Midline sagittal images obtained by lumbar T2-weighted magnetic resonance imaging were used to evaluate disc degeneration. Participants with one or more degenerated discs were classified into the disc degeneration group. A 2000 m race trial using a rowing ergometer was conducted. Surface electrodes were attached to the right rectus abdominis, external oblique, internal oblique, latissimus dorsi, multifidus, erector spinae, rectus femoris, and biceps femoris. The activity of the muscles was measured during one stroke immediately after 20% and 80% of the rowing trial. Nonnegative matrix factorization was used to extract the muscle synergies from the electromyographic data. To compare the muscle synergies, a scalar product (SP) evaluating synergy coincidence was calculated, and the muscle synergies were considered identical at SP > 75%. Both groups had only one module in the 20% and 80% time points of the trial. At the 20% time point of the 2000 m rowing trial, the SP of the module was 99.8%. At the 80% time point, the SP of the module was 99.9%. The SP results indicate that, at 20% and 80% time points, both groups had the same module. The module showed a high contribution in all muscles. The activation coefficients indicated that the module was always highly activated throughout the rowing stroke in both groups. The trunk and lower extremity muscles are mobilized through the rowing stroke and maintain coordination during rowing. There was no difference in the muscle synergy between the rowers with and without lumbar intervertebral disc degeneration.

## 1. Introduction

The central nervous system controls movement through a combination of a few basic activation patterns known as motor modules or muscle synergies [1]. A muscle synergy can be characterized as a low-dimensional organizational structure controlling multiple muscles. The evaluation of muscle coordination was refined by nonnegative matrix factorization (NMF) analyses based on Bernstein's concept [1]. This analysis divides electromyographic (EMG) data into two factors: muscle weighting and activation coefficient. Muscle weighting represents the relative weighting of each muscle within each module, and the activation coefficient represents the relative activation of the muscle weighting [2].

Recently, using NMF analysis, muscle synergy in competitive sports has been analyzed. As a result, it is reported that the number of muscle synergy changes every sports activity and that muscle synergy differs by the performance level and existence of injury. For example, in the research which evaluated the muscle synergy during sidestepping, it was shown that groin pain causes motor control dysfunction of the trunk and lower extremity muscle groups [3]. Motor control of the upper and lower extremities and the trunk is very important in rowing. Therefore, it may be connected with injury prevention and performance improvement by clarifying the muscle synergy in rowing. Muscle synergy during rowing has been analyzed in experienced rowers and untrained subjects. In research comparing the muscle synergy between experienced rowers and untrained subjects during rowing at high stroke rates, three synergies were identified in both groups, confirming the similarity in muscle synergy between groups [4, 5]. In the study of collegiate rowers and recreational athletes with no rowing experience, three synergies were identified in both groups during rowing [6].

In terms of injuries to rowers, the lumbar spine is the most common site of injury [7–9]. Therefore, a number of studies on the factors contributing to low back pain (LBP) have been performed, and LBP history [10] and ergometer training [9, 11] have been reported as significant risk factors for LBP in rowers [12]. In addition, signs of disc degeneration are associated with LBP [13]. A longitudinal study that investigated the relationship between LBP and intervertebral disc degeneration in collegiate rowers also reported that lumbar intervertebral disc degeneration is related to LBP [14]. Therefore, in this study, we focused on lumbar intervertebral disc degeneration associated with LBP in rowers. A previous study involving combat sports athletes reported that the relative size of the cross-sectional areas of the trunk muscles to their body weight in the lumbar intervertebral disc degeneration group was significantly smaller than that in the nonlumbar intervertebral disc degeneration group [15]. Accordingly, it was thought that the trunk muscles are related to lumbar intervertebral disc degeneration. As described above, motor control of the upper and lower extremities and the trunk is very important in rowing. Therefore, we hypothesized that the rowers developing intervertebral disc degeneration might have different muscle coordination of the trunk and lower extremities while rowing, as compared to those who did not develop any intervertebral disc degeneration. Rowers with disc degeneration may have motor control dysfunction during rowing, but muscle synergy during rowing has not been compared in rowers with and without lumbar intervertebral disc degeneration.

Therefore, this study is aimed at clarifying the trunk and lower extremity muscle synergy during rowing and at comparing the muscle synergy between elite rowers with and without lumbar intervertebral disc degeneration.

## 2. Materials and Methods

### 2.1. Participants

The study participants were 12 elite collegiate rowers with career durations of >3 years, including six rowers with lumbar intervertebral disc degeneration (sex: male, *n* = 4; female, *n* = 2; age: 19.8 ± 0.8 years; body mass index: 21.7 ± 1.3 kg/m^2^; and duration of rowing career: 5.1 ± 2.2 years) and six rowers without lumbar intervertebral disc degeneration (sex: male, *n* = 4; female, *n* = 2; age: 21.2 ± 0.8 years; body mass index: 23.3 ± 1.5 kg/m^2^; and duration of rowing career: 6.5 ± 2.0 years). All participants belonged to the same university team. Their training involved mainly rowing for approximately 11 sessions a week for approximately 2 hours per session, which included weight training approximately twice a week. The experiment was carried out according to the tenets of the Declaration of Helsinki. This study was approved by the institutional ethics review committee (approval number: 2012-223). All participants provided informed consent to participate in this study.

### 2.2. Experimental Protocol

A 2000 m rowing trial was conducted using a Concept 2 Model D rowing ergometer (Concept Inc., Morrisville, VT, USA). The warm-up was performed on land and included ergometer rowing, with similar intensity and duration among the participants. After warming up, electrodes and a wireless EMG system were attached to the participants. As in previous studies that investigated the kinematics and kinetics of rowing [16, 17], participants were asked to row at a race pace.

### 2.3. Assessment of Disc Degeneration

Lumbar T2-weighted sagittal magnetic resonance (MR) images (repetition time: 2800 ms; echo time: 90 ms) were obtained using a 1.5-T MR device (Signa HDxt XV; GE Healthcare, Tokyo, Japan) with a four-channel spine coil. The slice thickness was 4.0 mm, and the field of view was 300 × 300 mm. The midsagittal image was used for the evaluation. Using the Pfirrmann classification [18], the L1–L2 to L5–S1 discs were classified into five grades according to the degree of degeneration. Participants with one or more degenerated discs were classified into the disc degeneration group. Degeneration was assessed by two experienced orthopedic surgeons. MR images were obtained approximately 4 months before the rowing ergometer task because disc degeneration was assessed retrospectively.

### 2.4. Data Measurements

Muscle activity was measured using a wireless EMG system (EMG-025; Harada Electronic Industry Ltd., Sapporo, Japan) at a sampling frequency of 983.217 Hz. Before the surface electrodes were attached, skin abrasives and alcohol were applied to the skin to achieve an electrical resistance of ≤2 k*Ω*, and pairs of disposable Ag/AgCl surface electrodes (BlueSensor N-00-S; Ambu, Ballerup, Denmark) were attached parallel to the muscle fibers, with a center-to-center distance of 2 cm. Surface EMG data were collected from the right rectus abdominis (3 cm lateral to the umbilicus) [19, 20], external oblique (15 cm lateral to the umbilicus) [21], internal oblique (the abdominal muscle corresponding to two fingerbreadths medial to the anterior superior iliac spine), multifidus (2 cm lateral to the L5 spinous process) [22], erector spinae (3 cm lateral to the L3 spinous process) [19, 20], latissimus dorsi (the belly muscle corresponding to three fingerbreadths inferior to the posterior axillary fold) [23], rectus femoris (the point corresponding to 50% of the distance between the anterior superior iliac spine and the upper margin of the patella) [23], and biceps femoris (the point corresponding to 50% of the distance between the head of the fibula and the ischial tuberosity) [23]. A reference electrode was placed over the sternum. To divide the rowing cycle, a digital video camera (Exilim EX-FH25; Casio Computer Co., Ltd., Tokyo, Japan) synchronized with the EMG system was used to make a recording at 29.97 frames per second. Reflective markers with a diameter of 19 mm (QPM190; Qualisys, Gothenburg, Sweden) were attached to the left side of the handle and the seat.

### 2.5. Data Analysis

The time point at which the *x*-coordinate of the sheet marker increased was referred to as the trial starting point. The *x*-coordinate determined where the point was in a left-right direction. The catch position was defined as the time at which the *x*-coordinate of the handle marker showed the minimum value. The time between the catch position and the next stroke's catch position was referred to as the stroke (one rowing cycle, Figure 1). The marker coordinates were defined using DIPP-Motion Pro (Ditect Co., Ltd., Tokyo, Japan).

A custom MATLAB (MATLAB R2016; MathWorks, Inc., Natick, MA, USA) code was used on the linear envelope and NMF. EMG data (raw data) corresponding to one rowing cycle were extracted. The EMG data were normalized to the maximum value of the EMG amplitudes over all conditions within the same participant for each muscle. Thus, the EMG scales ranged from 0 to 1. The rectified EMG signals were transformed into the linear envelope. One stroke at the 20% time point and another at the 80% time point of the 2000 m rowing trial were analyzed. To normalize time, the rowing cycle was interpolated to 101 time points. NMF was then performed to extract muscle synergies as described by Lee and Seung [24], using the following formulas:

(1) $$\begin{array}{c} E=WC+e, \end{array}$$

(2) $$\begin{array}{c} \underset{\begin{array}{c} W>0\\ C>0 \end{array}}{\min}{\left|\left|E-WC\right|\right|}_{\text{FRO}}, \end{array}$$

where *E* is a *p* × *n* initial matrix (*p* is the number of muscles, and *n* is the number of time points) that represents the EMG matrix. The initial matrix *E* consisted of a cycle for each of the eight muscles; therefore, *E* was a matrix with 8 rows and 101 columns. *W* is a *p* × *s* matrix (*s* is the number of synergies) that represents the muscle weighting. *C* is an *s* × *n* matrix that represents the activation coefficient, and *e* is a *p* × *n* matrix that represents the residual error matrix. Equation (2) indicates that matrix *e*, calculated using Equation (1), reaches a minimum. For each participant, we iterated the analysis by varying the number of synergies between 1 and 8. We selected the least number of synergies that accounted for >90% of the global variance accounted for (VAF) [2, 25, 26] and >75% of the local VAF [2]. Based on these studies, global and local VAFs were calculated as follows:

(3) $$\begin{array}{c} \text{Global VAF}=\left(1-\frac{\sum_{i=1}^{p}\sum_{j=1}^{n}\;{\left(e_{i,j}\right)}^{2}}{\sum_{i=1}^{p}\sum_{j=1}^{n}\;{\left(E_{i,j}\right)}^{2}}\right)\times 100\;\left(\%\right), \end{array}$$

(4) $$\begin{array}{c} \text{Local VAF }\left[\text{m}\right]=\left(1-\frac{\sum_{j=1}^{n}\;{\left(e_{m,j}\right)}^{2}}{\sum_{j=1}^{n}\;{\left(E_{m,j}\right)}^{2}}\right)\times 100\;\left(\%\right), \end{array}$$

where *i* ranges from 1 to *p* and *j* ranges from 1 to *n*. Thus, in this study, *i* ranged from 1 to 8 and *j* ranged from 1 to 101. In Equation (4), *m* represents the muscle “m.”

### 2.6. Statistical Analysis

A scalar product (SP), calculated according to the formula described by Cheung et al. [27], compared the synergies between the groups with and without disc degeneration. We defined the module as the same if the SP was >75%.

(5) $$\begin{array}{c} \text{SP}=\frac{\vec{W_{\text{degeneration}}}\cdot \vec{W_{\text{normal}}}}{\left|\vec{W_{\text{degeneration}}}\right|\left|\vec{W_{\text{normal}}}\right|}\times 100\;\left(\%\right), \end{array}$$

where each $\overset{⃑}{W}$ is the averaged vector among the participants in each group and $\vec{W_{\text{degeneration}}}$ and $\vec{W_{\text{normal}}}$ are the $\overset{⃑}{W}$ of the groups with and without degeneration, respectively. SP were performed using a custom MATLAB (MATLAB R2016; MathWorks, Inc., Natick, MA, USA). Other statistics were performed using SPSS version 27.0 (IBM Corp., Armonk, NY, USA), and statistical significance was set at *p* = 0.05. Unpaired *t*-tests were conducted for the two groups (with disc degeneration vs. without disc degeneration) for rowing stroke ratings at the 20% and 80% time points and 2000 m rowing time. The Kolmogorov-Smirnov test was conducted to confirm the normality of the data. As a result of the normality test, parametric testing was selected.

## 3. Results

Table 1 shows the results of the performance data. The rowing stroke ratings at the 20% time point were 29.4 ± 2.4 strokes per minute and 29.1 ± 2.3 strokes per minute for the disc degeneration group and nondisc degeneration group, respectively (*p* = 0.81). The rowing stroke ratings at the 80% time point were 29.6 ± 1.5 strokes per minute and 29.8 ± 2.0 strokes per minute for the disc degeneration group and nondisc degeneration group, respectively (*p* = 0.84). The 2000 m rowing times were 440.9 ± 29.4 seconds and 432.2 ± 33.3 seconds for the disc degeneration group and nondisc degeneration group, respectively (*p* = 0.64). The rowing stroke ratings and 2000 m rowing time did not show any significant differences between the two groups.

Figure 2 shows the EMG data of the mean of the two groups during a rowing stroke.  Table 2 and Figure 3 show the results of the NMF analysis. At both the 20% and 80% time points of the 2000 m rowing trial, when there was one module, the global and local VAFs exceeded 90% and 75%, respectively, for the first time (Table 2). Therefore, one module was extracted in each group (Figure 3). All participants had one module. At the 20% time point of the 2000 m rowing trial, the SP of the module was 99.8%. At the 80% time point, the SP of the module was 99.9%. The SP results indicate that, at 20% and 80% time points, both groups had the same module. In both the 20% and 80% time points, the data from the module mainly reflected that all muscles have high degrees of contribution. The activation coefficients indicated that the module in both groups was always highly activated throughout the rowing stroke, even during the recovery. There was no significant difference between the groups with and without disc degeneration.

## 4. Discussion

This study investigated eight muscles functioning during a 2000 m rowing trial and compared their activities between the rowers with and without disc degeneration. The main findings of this study were that only one module was active at the 20% and 80% time points of the 2000 m rowing trial, and there was no significant difference between the groups with and without disc degeneration. The module showed a high contribution in all muscles, and the activation coefficients indicated that the module was highly activated throughout the rowing stroke in the groups with and without disc degeneration. Therefore, it is suggested that the trunk and lower extremity muscle groups are mobilized through the rowing stroke and maintain coordination during the rowing motion.

Turpin et al. [28] analyzed the muscle synergy during rowing in nine male participants who had no prior experience in rowing and reported that there was no change in the number of synergies during the fatiguing rowing test. In their study, subjects performed the fatiguing rowing test for up to 6 minutes, and the amount of power required increased every 2 minutes. In our study, there was no difference in the number of synergies during the 2000 m rowing trial, and the result was similar to that of the previous study. On the other hand, it has been reported that antagonistic muscle prefatigue led to significantly lower gamma-band corticomuscular coherence during an isometric elbow extension, and muscle fatigue may reduce coherence [29]. In this study, we did not examine the difference in muscle fatigue between the 20% and 80% time points, but corticomuscular coherence may have been reduced at the 80% time point. The number of modules in various athletic movements has been investigated, and it has been reported that Japanese archery has two modules [30], and running has four modules [31]. Muscle synergies have also been investigated in swimming; underwater undulatory swimming and breaststroke swimming have three modules [32, 33]. Unlike other sports that consist of multiple modules, the results of this study suggest that rowing does not require multiple modules. On the other hand, previous studies investigating muscle synergy during rowing have detected three synergies [4–6]. In previous studies, 16 to 23 muscles, including upper extremity muscles, were analyzed, but in this study, only 8 muscles were included in the analysis. The small number of test muscles compared to that in the previous study may have influenced the result of only one synergy in this study.

In our study, we focused on the lumbar intervertebral disc degeneration in elite rowers and found no difference in the muscle coordination between the groups with and without disc degeneration. It is possible that there was no significant difference in muscle synergy between the two groups because the presence of LBP in both groups was not considered in this study. Since disc degeneration becomes a factor of LBP, rowers with disc degeneration may experience LBP during rowing, which may affect their coordination. However, it is not clear whether the subjects with disc degeneration had LBP at the time of the rowing trial, and thus, there may have been no difference in muscle synergy between the two groups. In addition, in our study, the disc degeneration grade was a grade 3 or 4 with no participants having the most advanced disc degeneration (grade 5). The subjects had one or two degenerated discs. If the subjects had many degenerated discs or the degree of degeneration was more severe, there might have been differences in muscle synergy between the two groups.

The limitations of this study were that the upper extremity muscles were not measured and that the number of analyzed muscles may be insufficient. Therefore, the upper extremity muscles should be included in future investigations. In addition, the existence of LBP was not considered in this study. Therefore, further investigations considering the existence of LBP are necessary for the future.

## 5. Conclusions

In conclusion, all the muscles have high contributions in the single model during rowing. The activation coefficients indicate that the module is highly activated throughout the rowing stroke, and there is no difference in the muscle synergy between rowers with and without lumbar intervertebral disc degeneration.

## Figures and Tables

**Figure 1:** One rowing cycle. The catch position was defined as the time at which the *x*-coordinate of the handle marker showed the minimum value. The time between the catch position and the next stroke's catch position was referred to as the stroke (one rowing cycle).

**Figure 2:** EMG data of the mean of the two groups during a rowing stroke. The DD group is the group with disc degeneration. The non-DD group is the group without disc degeneration. The EMG scales ranged from 0 to 1. Solid line: 20% time point of the 2000 m rowing trial; dashed line: 80% time point of the 2000 m rowing trial. DD: disc degeneration; EMG: electromyographic.

**Figure 3:** Extracted module during the 2000 m rowing trial. SP indicates the similarity between the groups with and without disc degeneration. RA: rectus abdominis; EO: external oblique; IO: internal oblique; MF: multifidus; LD: latissimus dorsi; ES: erector spinae; RF: rectus femoris; BF: biceps femoris; SP: scalar product.

**Table 1:** Results of the performance data.

	DD group	non-DD group	*p* value
Rowing stroke ratings (20%) (strokes per minute)	29.4 ± 2.4	29.1 ± 2.3	0.81
Rowing stroke ratings (80%) (strokes per minute)	29.6 ± 1.5	29.8 ± 2.0	0.84
2000 m rowing time (seconds)	440.9 ± 29.4	432.2 ± 33.3	0.64

The DD group is the group with disc degeneration. The non-DD group is the group without disc degeneration. The performance data did not show any significant differences between the two groups. DD: disc degeneration.

**Table 2:** Results of the nonnegative matrix factorization analysis (number of modules = 1).

		20% time point	80% time point
Global VAF (%)		98.1 ± 2.6	98.6 ± 1.7

Local VAF (%)	RA	83.2 ± 11.2	79.0 ± 20.5
	EO	83.6 ± 10.9	80.3 ± 20.2
	IO	82.3 ± 12.2	78.1 ± 20.8
	MF	84.9 ± 10.3	80.4 ± 20.1
	LD	84.4 ± 10.6	79.5 ± 21.0
	ES	84.2 ± 10.7	81.1 ± 20.4
	RF	83.2 ± 11.8	79.2 ± 21.3
	BF	83.9 ± 10.5	80.2 ± 20.4

VAF: variance accounted for; RA: rectus abdominis; EO: external oblique; IO: internal oblique; MF: multifidus; LD: latissimus dorsi; ES: erector spinae; RF: rectus femoris; BF: biceps femoris. VAF corresponding to the number of modules. The number of modules is decided when the global VAF exceeds 90% and the local VAF exceeds 75% for the first time.

## Data Availability

The datasets analyzed during the current study are available from the corresponding author on reasonable request.
